RETRACTED

# A Novel English Translation Model in Complex Environments Using Two-Stream Convolutional Neural Networks

**DOI:** 10.1155/2022/8426460

**Published:** 2022-09-05

**Authors:** Lijuan Zhang

**Affiliations:** Shanghai Jian Qiao University, Shanghai 201306, China

## Abstract

Although translation is an essential component of learning English, it does not receive the attention it merits in the modern English classroom. Teachers and students primarily emphasize listening, reading, and writing while neglecting the development of translation skills. The English test in China now reflects the fact that there are now very specific requirements for students' translation skills. As a result, we should emphasize developing students' translation skills when teaching them English. The following experimental data can be obtained following the study and experiment on the English translation simulation model based on the two-stream convolutional neural network: English vocabulary and grammar have passing and excellent rates of 90 and 57 percent, respectively, while reading has passing and excellent rates of 69 and 8 percent, respectively. The ability of students to translate into English has significantly improved after using the English translation simulation model based on the two-stream convolutional neural network.

## 1. Introduction

A Chinese translation has been around for a while, and it has gone through the following stages of development. The study of Western translation theory began in the late Ming and early Qing dynasties, and the translation process reached the stage of in-depth research in the late Qing and early Ming dynasties, from the Southern Song Dynasty to the Sui and Tang Dynasties. After a considerable amount of time, translators started to focus on the translation of new literature, and after the rise of New China, translation studies expanded and became more thorough. Many translators have given up translating great Tibetan works in favor of other disciplines like mechanics, philosophy, biomedicine, astronomy, and mathematics due to the need to comprehend Western culture. Chinese translation advanced during the late Qing Dynasty and the early Republic of China, and numerous works were translated during this time. Numerous patriots put in a lot of effort during a time of national crisis to learn different Western translation theories and disseminate cutting-edge Western scientific and cultural knowledge, which not only helped to cultivate many Chinese scientific and technological talents but also gave western translation education a significant place in the history of modern Chinese translation.

For English majors, translation is a required course. China must develop outstanding translators who can adapt to various levels immediately in the age of globalization and information technology. The social responsibility of translation education cannot be ignored. The accumulation of history and Western theories over the past 30 years has greatly advanced translation education. Due to the unique nature of Chinese students learning English, translation remains a significant challenge in China. In order to accomplish this goal and raise the standard of translation instruction in schools, teaching methods must be given careful consideration in addition to student translation.

RETRACTED

Many English instructors and students put all of their attention into studying for exams and neglect translation. Giving pupils the chance to gain proficiency in translating can enhance their knowledge and influence learning in other subjects. Exams are so stressful that only grammar, composition, and other practical aspects are highlighted, and teachers' instructional priorities prevent the translation from becoming a part of actual learning. Teachers are exam-focused and motivated to educate students that they need to memorize vocabulary as well as numerous set phrases, sentence patterns, and specific formation patterns. They do not even believe that translation will boost students' English scores. Students find it challenging to translate, and some believe that translating does not help them to better their English. The effect of translation on the acquisition of English is nuanced rather than immediate. Many teachers and students do not think of or use translation in regular English classes because they do not see it as a way to enhance English learning. To address these issues, a two-stream convolutional neural network-based English translation simulation model is investigated in this research.

## 2. Related Work

This article studies some techniques of the English translation simulation model of the cloud dual-stream convolutional neural network, which can be fully applied to the research in this field. Najjar et al. explored the use of hyperbole in the Qur'an and its English translation, and they studied the morphological transformation of hyperbolic patterns [1]. Fitriani studied the syntactic and lexical aspects of the description and classification of grammatical errors found in English-translated sentences [2]. Yuval and Avishai described an optimization model based on dynamic programming and a public transport simulation that validates the benefits of such a model [3]. The elastic demand relationship that Shiaau and Wang embedded in the simulation model is used to estimate the impact of changing service time and lock-in during the simulation process [4]. These methods provide some references for our research, but they have not been recognized by the public due to the short time and small sample size of the relevant research.

RETRACTED

Based on the cloud dual-stream convolutional neural network, we have read the following related materials to optimize the English translation simulation model. Fang et al. proposed a novel multimodal biometric recognition system based on noncontact multispectral finger images, aiming to address the limitations of single-modal biometric recognition [5]. Li et al. proposed a real-time online gray-hot tracking method via Laplacian sparse representation in a Bayesian filtering framework [6]. Wu et al. proposed an infrared human action recognition method based on the spatiotemporal two-stream convolutional neural network [7]. Li et al. argued that the representational power of convolutional neural network (CNN) models for hyperspectral image (HSI) analysis is actually limited by the available number of labeled samples, which is usually insufficient to sustain deep networks with many parameters [8]. Xu et al. introduced a new model, the Regional Convolutional 3D Network (R–C3D), which uses a 3D fully convolutional network to encode the video stream, then generates candidate temporal regions containing activities, and finally classifies the selected regions as specific activity [9]. Ko and Chen believed that neural network manipulation systems were obtained by fitting data generated from optimal manipulation simulations [10]. Goh considered neural networks to be information processing systems whose architecture basically mimics the biological system of the brain [11].

## 3. Method for English Translation Simulation Model of Two-Stream Convolutional Neural Network

Exchanges between English and Chinese have increased as China's national power has grown, drawing attention from all around the world. Greetings are an essential part of everyday language use and cannot be disregarded. The foundation for the implementation of improved English translation education is the research of the two-stream convolutional neural network English translation simulation model.

### 3.1. Algorithms of Convolutional Neural Networks

Convolution layer calculation: The convolution layer calculation is to perform convolution multiplication between the input feature map vector and the convolution kernel, and the result of the convolution multiplication is transformed by the excitation function to obtain a new feature map. Due to the different convolution kernels, the feature maps obtained by different convolution kernels are also different. The feature map of each output is obtained by the combined convolution operation of multiple feature maps in the previous layer. The calculation of the convolutional layer is as follows:
  (1) $$\begin{array}{c} M_{j}^{l}=f\left(\sum_{i\in X_{j}}M_{i}^{l-1}*K_{ij}^{l}+b_{j}^{l}\right). \end{array}$$
In convolutional neural networks, the dominant excitation function is the sigmoid function, and each output function graph has a corresponding discriminant function. However, the convolution kernel for each function graph is the same [12].
Calculate the gradient of the convolutional layer: The convolutional layer *l* is usually followed by a sublayer *l* + 1, and the local feature of the convolutional layer feature map corresponds to a point in the sublayer feature map.
For each convolutional layer *j*, the error signal *δ*_*j*_^*l*^ of the feature map of the convolutional layer is given by:
  (2) $$\begin{array}{c} \delta_{j}^{l}=\beta_{j}^{l+1}\left(f^{\prime }\left(u_{j}^{l}\right)\cdot \text{up}\left(\delta_{j}^{l+1}\right)\right). \end{array}$$
Formula (2) represents the upsampling operation.
The bias basis gradient can be determined by summing the error signals of layer *l* using the above formula, as follows:
  (3) $$\begin{array}{c} \frac{\partial A}{\partial K_{ij}^{l}}=\sum_{u,v}{\left(\delta_{j}^{l}\right)}_{uv}{\left(p_{i}^{l-1}\right)}_{uv}. \end{array}$$
Since there are many weights in common in convolutional neural networks, the gradient of a given weight must be summed over all weights associated with that weight, and finally, its gradients are summed [13].
Calculation of downsampling layer: The principle of downsampling is that the size of each output function graph is a reduced version of the input function graph, as shown in the following formula:
  (4) $$\begin{array}{c} M_{j}^{l}=f\left(\beta_{j}^{l}\text{down}\left(M_{j}^{l-1}\right)+b_{j}^{l}\right). \end{array}$$
In the formula, down(·) represents the downsampling function; *β* represents the multiplicative bias parameter; *b* represents the additive bias parameter.
The size of the downsampling window is *y* ∗ *y*, so the graph of the output function is reduced by a factor of *y*. The purpose of downsampling is to reduce the resolution for scaling invariance. Each output graph has its own multiplication and addition difference parameters.
Calculation of the downscaling gradient: To calculate the error signal for the sensitivity map of the downscaled layer, one must first locate the layer that corresponds to the pixel in the sensitivity map of the current layer. Then, one must recursively calculate the current error signal using the error signal of the subsequent layer, as shown in the following formula:
  (5) $$\begin{array}{c} \delta_{j}^{l}=f^{\prime }\left(u_{j}^{l}\right)\cdot \text{conv}2\left(\delta_{j}^{l+1},\text{rot}180\left(K_{j}^{l+1}\right),“\text{full}”\right). \end{array}$$

Among them, full represents the full convolution function [14].

RETRACTED

“Full” is a full convolution function that processes and analyzes convolution gates, replacing missing pixels with 0 s, so *β* and *b* can be determined. This can be illustrated by the following formula:

(6) $$\begin{array}{c} \frac{\partial A}{\partial b_{j}}=\sum_{u,v}{\left(\delta_{j}^{l}\right)}_{uv},\\ \frac{\partial A}{\partial \beta_{j}}=\sum_{u,v}{\left(\delta_{j}^{l}\cdot \text{down}\left(M_{j}^{l+1}\right)\right)}_{uv}. \end{array}$$

Neurons are connected through axons, transmit signals through bulges, and adjust their states according to the “all or nothing” principle, that is, there are only two states. When the state of the neuron exceeds a certain threshold, it will be in the excited state, otherwise it will be in the inhibitory state.

Artificial neuron simulates biological neuron generation as the basic unit of convolutional network, which accepts input signal and generates certain output according to the set function. The basic structure of neurons is shown in Figure 1.

The neuron will receive *b* inputs *x* = (*x*_1_, *x*_2_,…, *x*_*n*_), and the input *y* can be expressed as the following formula:

(7) $$\begin{array}{c} y=f\left(\omega x+\omega_{0}\right), \end{array}$$

*b* represents the threshold, *f* (.) is the activation function, and *y* is the output component. Here, net_*j*_ represents the activation of the neuron unit, *x*_*i*_ represents the input of the unit, and *a*_*ij*_ represents the weight corresponding to each input, then the above relationship can be expressed by the following formula:

(8) $$\begin{array}{c} {\text{net}}_{j}=\sum_{i=1}^{n}a_{ij}x_{i}+b. \end{array}$$

Among them, *ω* = (*ω*_1_, *ω*_2_,…, *ω*_*n*_) is the n-dimensional weight, and *f* is the activation function. In order to enhance the function of the network, neurons need to introduce a variety of transfer functions. The commonly used transfer functions are:

(9) $$\begin{array}{c} f\left(s\right)=\left\{\begin{array}{c} r,\;s>r,\\ s,\;s\leq r,\\ -r,\;s<-r. \end{array}\right. \end{array}$$

In the neural network, *r* and −*r* are the thresholds. If *s* is greater than *r*, the neuron outputs *r*. If *s* < −*r*, the neuron outputs −*r*, and the other outputs are *s*.

Sigmoid function, Sigmoid is an *S*-shaped nonlinear activation function, and its expression is as follows:

(10) $$\begin{array}{c} y=f\left(s\right)\\ =\begin{array}{c} 1\\ 1+c^{-s} \end{array}. \end{array}$$

Sigmoid neurons and perceptron neurons are basically the same, which can make the output results slightly change when the weights change slightly. The input of the function can be classified into the range of 0 to 1, and the middle area is gained, and the two sides are suppressed. When *s* is a large negative number, the output is approximately 0, and when *s* is a large positive number, the output is approximately 1.

RETRACTED

The hyperbolic tangent function, hyperbolic tangent function can be regarded as a translated and enlarged Sigmoid function, and its expression is as follows:

(11) $$\begin{array}{c} f\left(s\right)=\begin{array}{c} c^{s}-c^{-s}\\ c^{s}+c^{-s} \end{array}\\ =2*Sig\mathrm{mod}\left(2s\right)-1. \end{array}$$

Unlike the sigmoid function, the hyperbolic tangent function has a mean of 0. The hyperbolic tangent function has better performance in image processing applications.

In recent years, Convolutional Neural Networks (CNN) have become the focus of machine learning research [15]. In 1986, the BP algorithm was introduced, which laid the foundation for CNN. In 2012, CNN won the ILSVRC competition. Since then, CNN has been applied in many fields.

Currently, there are two main approaches to action recognition using convolutional neural networks. One is a 3D Convolutional Neural Network, which uses ordered video images as the input to the network. The other is a two-stream convolutional neural network using post fusion, which is based on the fusion of two separate recognition streams, the spatial stream and the temporal stream [16]. Both streams are based on the combination of two-stream structure and 3D convolution to propose a spatiotemporal convolutional neural network structure, which is a breakthrough achievement.

Two-stream network structure Each stream applies a convolutional neural network. The basic structure of the convolutional neural network is shown in Figure 2.

The output features of the two streams are fused and then entered into the classifier for behavior classification and recognition. The input of this network structure is a block of stacked *L* frames, and the input of the temporal stream and the spatial stream are also different. The input to the spatial stream is a single frame, and this stream effectively identifies actions from static frames because some actions are closely associated with specific objects. The input of the temporal stream is the stacked optical flow displacement field of several consecutive frames. Optical flow accurately extracts dynamic features between frames, which makes actions easier to recognize. The static and dynamic features of the action are extracted by CNN and then combined in the fusion layer. The action features extracted in this way have both specific attributes on a single frame and temporal associations, so that classification and recognition tasks will have better results. And then these features are sent to the classifier to obtain the classification result.

RETRACTED

Fusion can be applied at any layer in the two networks, which requires the feature maps of the two networks to have the same spatial dimension at time *t*, which can be achieved using up-convolution or upsampling. Based on the recognition accuracy obtained from the split1 dataset of UCF101, both spatial and temporal streams adopt the AlexNet structure [17]. The effect of different fusion positions on the accuracy is shown in Figure 3.

As can be seen from Figure 3, the recognition accuracy obtained by fusion at different layers, it can be clearly seen that the fusion accuracy after conv5 is higher. And since it is fused before the fully connected layer, the number of parameters is twice less than that in the softmax layer. The effects of different fusion methods on the accuracy are shown in Table 1.

Table 1 shows the performance of different fusion methods, which can make the convolution fusion method work best, and the recognition rate of the fusion layer using the combination of 3D convolution and 3D pooling is improved. The reason why it is fused after the conv5 layer is because of the correspondence between the spatial static image features and the changing features of the action, and the fusion of spatial and temporal information, while the features of the fully connected layer lack such characteristics.

The results show that the fusion needs to learn fewer parameters before the fully connected layer, and the model performance is better. A fusion layer is added after the last convolutional layer, and the input of the fusion layer is the feature maps of the two streams. The network uses the AlexNet network, which is currently widely used in behavior recognition tasks to fuse at the ReLU5 layer (that is, the activation layer after Conv5), and then input the fully connected layer to obtain the loss, and then obtain the gradient according to the loss function, backpropagation, so as to optimize the parameters in the network [18].

### 3.2. English Translation

The accuracy and reliability of translations are frequently in conflict due to the significant differences between Chinese and English. Consequently, in order to avoid awkward and rigid translations, it is essential when translating to understand the differences in idioms and semantics between the two languages.

For sentence pattern selection, we must first understand the differences between English and Chinese language structures. Chinese prose emphasizes the physical and spiritual gathering, while English prose emphasizes the internal logical relationship between sentences. The Chinese structure is loose and the English structure is strict. English sentences have important connectives under them, while Chinese sentences use few or no connectives but are still fluent. For this reason, linguists often use bamboo syntax to compare English sentences and running water syntax to compare Chinese sentences. However, Chinese and English sentences also have many similarities, which also provides convenience and possibility for translation [19].

RETRACTED

The difficulties posed by cultural differences must also be taken into account when translating; it is not just a matter of language. The domestication method and the transfer method are two approaches to dealing with the cultural aspects of the text, i.e., home to the culture of the source language and home to the culture of the target language. The various translation goals, the text's type, the author's intended audience, and the chosen method must all be considered by the translator.

Compared with literary English, technical English has linguistic peculiarities, especially in terms of vocabulary and syntax. The first is the use of a broad range of technical terms, including purely scientific and technical terms, general scientific and technical terms, and semi-technical terms, i.e., terms that have a common meaning in themselves but have different meanings in different disciplines and fields. The second is to use abbreviations, and again, there are more nouns or noun phrases. Therefore, in the specific translation process, for the processing of vocabulary, it is necessary to consult a lot of materials and try to figure out the original text, especially the professional connotation of general vocabulary, so as to achieve lexical equivalence. In terms of syntax, English for Science and Technology uses more passive voice, complex structures, and various clauses to reflect objective and accuracy and avoid subjective narration. The syntax of technical English can be said to be “complicated in structure, many layers, indistinguishable, too many episodes, difficult to find context, reversed word order, and distorted structure.” Therefore, in the translation process, it is not enough to achieve lexical equivalence. It is also necessary to correctly understand the original text at the syntactic level, clarify the sentence structure, and on this basis, pay attention to morphological modifications and adjust the word order to correctly convey information.

The main function of technical English is to convey information. In other words, technical English translation also means conveying information and improving technical communication. Some scholars define translation as “achieving the best possible equivalence between text in the target language and text in the source language, first semantically and secondly stylistic equivalence.” Therefore, this equivalence must also be achieved in technical English translation [20].

RETRACTED

According to the functional equivalence theory, the dynamic relationship between the source and target languages is more significant to the translator than a direct correspondence. In other words, the relationship between the person receiving the translation and the information being translated should, in theory, be the same as the relationship between the person receiving the information being translated and the information being originally translated. Content is prioritized over form according to the functional equivalence theory, which emphasizes that both the original text's author and the target language readers can come to a mutual understanding and appreciation as well as dynamic equilibrium. In this procedure, the translator is crucial. Repeated thought and precise application of translation techniques are required to accurately reproduce the original author's ideas. In technical English translation, the lexical equivalence strategy is crucial. An English sentence should typically have two main components. The two main parts of a sentence are the subject and the predicate. Nouns and verbs make up the majority of the vocabulary in a sentence, and it's crucial that they match up consistently. The equivalence of the words that make up sentences, which can express various logical relationships, is also significant.

### 3.3. Simulation Model

Eigen Trust is a global trust-based model proposed in 2003. It is a typical reputation model, and many later reputation models are improved and perfected on the basis of it. In the Eigen Trust model, a node has a globally unique reputation value, which is calculated iteratively through the reputation evaluation of the entire network. The calculation of reputation is based on the trust transfer between nodes, and its calculation method is as follows:

(12) $$\begin{array}{c} T_{ak}=\sum_{b}C_{ab}*C_{bk}. \end{array}$$

The meaning of this calculation method is that when node a wants to know the reputation value of node *k*, it asks its neighbor node *b* to get its evaluation of node *k*. Then according to its own evaluation of *b* and b's evaluation of *k* to calculate its own evaluation of *k*.

In the above calculation formula, *C*_*ab*_ represents the local reputation value of node *a* to node *b*, and the calculation method is:

(13) $$\begin{array}{c} C_{ab}=\frac{\max\left(S_{ab},0\right)}{\sum_{b}\max\left(S_{ab},0\right)}. \end{array}$$

Sab represents the number of times that node *a* is satisfied with node *b* during the transaction between node a and node *b*. In this model, it is assumed that there will always be a fixed set of pretrusted nodes in the network. Due to the setting of the set, it is always possible to converge in the iterative calculation, and the nodes in the set all have high reputation values. But how to select the node set itself is a difficult problem to solve.

RETRACTED

SVM is a binary classification model based on maximizing intervals in the function space. Suppose someone is dealing with a binary classification problem, and a linear machine with reference vectors assumes that all elements in the input and output spaces match. SVM transforms training samples into a function space, generates a learned classifier, transforms test samples in the same way during testing, and uses the learned classifier to predict classes. Suppose there is a training dataset T:

(14) $$\begin{array}{c} T=\left\{\left(m_{1},n_{1}\right),\left(m_{2},n_{2}\right),\ldots ,\left(m_{Y},n_{Y}\right)\right\}. \end{array}$$

Among them,

(15) $$\begin{array}{c} m_{i}\in M,\;n_{i}\in N=\left\{+1,-1\right\},\;i=1,2,\ldots ,Y, \end{array}$$

*m*_*i*_ is the *i*th identification vector, *n*_i_ is the category of mi, if *n*_*i*_ = +1, it is one category, otherwise it is another category.

SVM aims to utilize hyperplanes to separate input data into two classes in feature space. In the general case of linearly distributed training data, there are infinitely many ways to split all the sample data. Therefore, linear support vector machines use the interval maximization criterion to find the best segmentation method, where the selected segmentation hyperplane is the only solution. The separation of the hyperplane is shown in Figure 4.

As shown in Figure 4, *H* is the optimal distribution hypergraph of linearly separable samples, and the pentagonal blocks and triangular blocks represent different sample data. *H*1 and *H*2 are the two distribution lines selected for the samples corresponding to the pentagon block and the samples corresponding to the triangles just divided, and the optimal distribution line *H* is located between *H*1 and *H*2. At this time, the interval between *H*1 and *H*2 is called a classification interval. The selection criterion of *H* is not only to separate the two types of samples as much as possible, but also to make the classification interval between *H*1 and *H*2 as large as possible. The objective function to solve the optimal separating hyperplane of SVM is:

(16) $$\begin{array}{c} \underset{w.r}{\min}\frac{1}{2}{\left\|w\right\|}^{2}\text{s.t.}l_{k}\left(w^{T}x_{k}+r\right)\geq 1,\;k=1,2,\ldots ,K. \end{array}$$

The solution of the optimal separating hyperplane can be solved by transforming formula (16) from the original problem to the dual problem using the algorithm of the Lagrangian dual problem. The objective function of formula (16) is transformed into:

(17) $$\begin{array}{c} D\left(u\right)=\mathrm{sgn}\left\{\left(w^{T}u\right)+\tilde{r}\right\}\\ =\mathrm{sgn}\left\{\sum_{k=1}^{K}b_{k}y_{k}\left(u_{k}u\right)+\tilde{r}\right\}. \end{array}$$

Among them, sgn is the symbolic function, *u u*_*i*_ is the dot product of *u* and *u*_*i*_, and *w*, *b*_*k*_, and *r* are the variables that share the hyperplane. In the case of linear inseparability, formula (16) can be transformed into:

(18) $$\begin{array}{c} \underset{w.\eta }{\min}\frac{1}{2}{\left\|w\right\|}^{2}+C\left(\sum_{k=1}^{K}\eta_{k}\right)\text{s.t.}l_{k}\left(w^{T}u_{k}+r\right)-1+\eta_{k}\geq 0,\;k=1,2,\ldots ,K. \end{array}$$

Among them, *C* > 0 is a constant to reduce the misclassification constraint and *η*_*k*_ is a relaxation term. The objective function in formula (18) is an expression of the trade-off between the maximum classification interval and the minimum number of misclassified samples.

RETRACTED

The development of IDS simulation model is essentially a special software development process. It is a typical network security detection equipment. The research of the IDS simulation model helps discuss and summarize the modeling method of the detection mechanism simulation model. Therefore, the idea of Model-Driven Framework (MDA) is introduced, and the modeling idea of the simulation model, the adopted modeling method, the structure of simulation model and the mapping relationship between models are described.

The detection mechanism is an important link in the model, which is the key to changing from static protection to dynamic response. Taking IDS as an example, the establishment and verification of the detection mechanism simulation model are studied. The corresponding simulation model needs to meet the following requirements:

1. To highlight functional modeling and simulation, the simulation model should reflect the functional essence of IDS. The simulation of the detection mechanism mainly focuses on the simulation of the function, and the focus is on whether the system can complete the expected detection function according to the set security policy during the simulation process.
2. The simulation model must be reusable, and the purpose of the detection mechanism modeling is not to meet a specific application but to adapt to the different needs of network security simulation.
3. The simulation model must be complete and effective, and a correct simulation model is a premise for the credibility of the simulation results. Therefore, in the process of model establishment, it is necessary to ensure the completeness and effectiveness of its functions by means of verification and other means.
4. The simulation model should have a flexible configuration interface to reflect the characteristics of intelligence; in the modeling process, human factors should be fully considered, and human reasoning and decision-making should be simulated through the detection rules to reflect its intelligent detection process.

RETRACTED

IDS is a complex system. Specifically, its complexity is mainly reflected in the following aspects. (1) The hierarchy of the architecture; (2) The complexity of information processing; (3) The uncertainty of system input and output information; (4) The intelligence of system behavior.

The development of modeling and simulation systems is essentially a special kind of software development process. The simulation model is finally embodied in the form of program code, and the establishment of the simulation model is also a special software development process. Therefore, Model-Driven Architecture (MDA), as a new software development framework, can also be used to guide the establishment of simulation models. The modeling process of the IDS simulation model is shown in Figure 5:

In Figure 5, there are five stages including requirements analysis, functional modeling, object modeling, program modeling, and model verification. (1) In the demand analysis stage, the simulation target of IDS and the specific requirements of the simulation model are mainly analyzed. (2) In the functional modeling stage, the IDS is essentially abstracted from the functional point of view, and the functional composition of the IDS is determined, as well as the restrictions and relationships between the various functions. (3) In the object modeling stage, based on the functional model, combined with the selected modeling platform, the platform-related object model is established through specific mapping rules. (4) In the program modeling stage, the object model is used as the input, and combined with the program modeling specification of the selected platform, the program model is established by automatic generation or manual writing. (5) Model verification stage. Model verification activities run through the above four stages, mainly to verify the correctness of the requirements document, functional model, object model, and program model generated in the modeling process to ensure the validity of the IDS simulation model.

RETRACTED

## 4. Experiment of English Translation Simulation Model of Two-Stream Convolutional Neural Network

### 4.1. Application Experiment of Convolutional Neural Network

In terms of resilience, self-learning capacity, and associative memory function, classical recurrent neural networks continuously imitate various brain functions. Artificial neural networks (ANNs) have a variety of network structures and functions. To ensure structural stability and design, it is necessary to integrate theoretical knowledge from various fields and disciplines, such as nonlinear and dynamical systems. As a result, it is crucial to research the structural design approaches used in recurrent neural networks. The block diagram of the recurrent convolutional neural network is shown in Figure 6.

As can be seen from the frame diagram of the recursive convolutional neural network, on the basis of the traditional convolutional neural network, after the network passes through the fully connected layer, it is not directed to the classification layer of the convolutional network, but directly to the added recurrent neural network layer. In this way, the results output by the recurrent neural network can be better applied in the classification layer.

The structure of the network is one more layer than the traditional convolutional neural network, and the complexity of the network is also improved. The learning algorithm of the recurrent convolutional neural network is mainly divided into two parts: one is the parameter adjustment in the convolutional neural network, and the other is the parameter training in the recurrent network.

In order to better verify and evaluate the performance of recurrent convolutional neural network, it is first applied to Chinese license plate recognition. This data set collects license plate figures from all over the country, divides them, and finally organizes them into a license plate data set. The network performance is tested on the commonly used dataset MNIST handwriting dataset. The dataset contains 60,000 training samples and 10,000 test samples. The test results of the license plate dataset are shown in Figure 7:

The three networks in Figure 7 are Convolutional Neural Networks, Elman Convolutional Neural Networks, and Elman-Jordan Convolutional Neural Networks. From the results in Figure 7, it can be seen that the Elman-Jordan convolutional neural network has a significantly lower error rate than the other two types of network models. It can be calculated from Figure 8 that the error rate of the recursive convolutional neural network for license plate testing is 41.27% lower than that of the convolutional neural network, and 11.24% lower than that of the Elman convolutional neural network. The test results on MNIST handwritten data are shown in Figure 8.

RETRACTED

From the data in Figure 8, it can be found that the error rate of the recurrent convolutional neural network for handwriting recognition has been reduced to a certain extent. Among them, it is 61.14% smaller than the convolutional neural network, and 21.06% smaller than the Elman convolutional neural network.

Overall, it can be said that the recurrent convolutional neural network has a lower error rate than the conventional convolutional neural network, which also demonstrates the recurrent neural network's superior classification capabilities. The recurrent convolutional neural network effectively utilizes this benefit of the recurrent network and improves the network's recognition capability. However, as the error rate decreases, the network's computation capacity grows as well, leading to more network iterations and an increase in the number of iterations overall, as well as an increase in the network's training time. This is due to the fact that the recurrent network recursively passes the network's output to the hidden layer so that it can take part in the network calculation. As a direct result, the network's parameters grow, which increases the network's overall computation.

### 4.2. Experiments on English Translation

The research objects are 33 full-time English translation students from a normal college in 2008. Use the CATTI Level 3 English Translation Comprehensive Ability Test to test the students' translation ability substantively. The translation method is English to Chinese. The structure of the test paper is shown in Table 2.

Vocabulary and grammar, reading, and cloze are three parts that make up this test paper. A maximum of 55 points can be awarded for the reading section. This shows that reading plays an important role in translation ability, it is the first process of translation work, and it is also the most basic prerequisite for doing a good job in translation work. The test was conducted with the help of 33 students and their teachers. The analysis of students' papers focuses on language skills (vocabulary, pragmatic skills, grammatical knowledge), the ability to modify sentence structure, reading skills and theory, and translation skills.

The overall average score for translation ability is 64.76, with the highest being 78.5 and the lowest being 42. The average score for translation management was 51.85, with the highest score being 67 and the lowest being 35. Of the 33 students, 6 passed the exam. The pass rate is 18.18%. This means that more than 80% of the students' translation skills do not meet the requirements of the CATTI syllabus. The results of each part of the translation are shown in Table 3.

RETRACTED

It can be seen from the table that the excellent rate and pass rate of the vocabulary and grammar part and the reading part are higher than those of the cloze part. The excellent and pass rates of the vocabulary and grammar sections were 57% and 90%, respectively, followed by the reading section, with a pass rate of 69%, but a lower excellent rate of 8%. And the most unsatisfactory cloze part, the pass rate is 32%, there is no excellent. Part of the reason for the low results is that the test is subjective, which makes the test more difficult. The results for each part are as follows:

1. Vocabulary selection, emphasizing the use of idioms, synonyms, analysis, and sentence comprehension.
2. Word replacement requires students to choose words or phrases that have similar meanings to the underlined part, mainly to check whether students understand the sentences and whether they are familiar with the concepts of “synonyms” and “synonyms.”
3. Proofread section covers the use of adjectives, nouns, common collocations, and an understanding of the meaning of major topics, while also examining grammar skills.

The second part: reading comprehension, which is the main part of translation work, consists of two reading articles. The first reflects the life and social status of black Americans, and the second is an article on popular science. The first reading score is shown in Figure 9.

The first reading was on sociocultural studies, and the results reflected in the papers showed that students had a good grasp of this cultural aspect, with 64% of them getting a distinction. The second reading score is shown in Figure 10.

The second reading mainly introduces the organic matter required for plant growth and its growth and development. As can be seen from Figure 10, translators have poor comprehension of technical articles, with only 10 students passing the test, 7 students getting good grades, and 6 received a failing grade. This suggests that liberal arts students have low scientific knowledge. Translation involves knowledge from all walks of life, and good translation requires the translator to have extensive knowledge.

## 5. Conclusions

Language proficiency is a crucial component of communicative language proficiency. It refers to the four fundamental abilities of listening, speaking, reading, and writing as well as the capacity to combine them. These four fundamental abilities combine to form translation, which is in essence a fundamental ability. Translation originally meant converting a text from one language to another. Oral and written translations between English and Chinese can be classified into two categories. The written translation reflects the students' “reading” and “writing” skills, whereas the oral translation reflects their “listening” and “speaking” skills. For advancing the current development of English translation, the research on the two-stream convolutional neural network-based English translation simulation model is also very important.

RETRACTED

## Figures and Tables

**Figure 1:** Basic structure of neurons.

**Figure 2:** Basic structure of a convolutional neural network.

**Figure 3:** The effect of different fusion positions on accuracy. (a) Fusion position accuracy 1. (b) Fusion position accuracy 2.

**Figure 4:** The optimal splitting hyperplane for the linearly separable case.

**Figure 5:** The modeling process of the IDS simulation model.

**Figure 6:** Structure diagram of recursive convolutional neural network.

**Figure 7:** Test results of license plate dataset.

**Figure 8:** Test results on MNIST handwritten data.

**Figure 9:** The first reading score.

**Figure 10:** The second reading score.

**Table 1:** Effects of different fusion methods on accuracy.

Integration methods	Fusion layer	Accuracy (%)
Max	Conv5	82.60
Sum	Conv5	85.10
2D conv	Conv5	85.86
3D conv + 3D pooling	Conv5	87.02

**Table 2:** The structure of the first volume of the CATTI English level 3 translator.

		Number of items	Scores	Time needed
Section 1	Vocabulary and grammar	50	25 points	2 hours
Section 2	Reading comprehension	50	55 points	
Section 3	Cloze	20	20 points	

**Table 3:** Proportion of achievements in each part of translation.

Ingredient/category	Vocabulary and grammar (%)	Reading ability (%)	Cloze ability (%)
Fail rate	10	31	68
Passing rate	90	69	32
Excellent rate	57	8	0

## Data Availability

The data used to support the findings of this study are included within the article.
